# Pathogenic Characterization of a Porcine Circovirus Type 3 Isolate from Heilongjiang, China

This article has been retracted.

**DOI:** 10.1155/2021/9434944

**Published:** 2021-06-24

**Authors:** Menghang Wang, Ying Yu, Jianan Wu, Fandan Meng, Yandong Tang, Shujie Wang, Yu Wang, Hongliang Cui, Xijun He, Yabin Tu, Gang Wang, Xuehui Cai

**Affiliations:** ^1^State Key Laboratory of Veterinary Biotechnology, Harbin Veterinary Research Institute, Chinese Academy of Agricultural Sciences, Harbin, China; ^2^College of Veterinary Medicine, Qingdao Agricultural University, Qingdao 266109, China

## Abstract

The clinical outcome of porcine circovirus 3 (PCV3) infection is still controversial. Herein, a novel PCV3 isolate (PCV3-China/DB-1/2017) with the molecular characterization of 24A and 27K in the Cap protein was used to inoculate three-week-old cesarean-derived, colostrum-deprived piglets. The nine PCV3 DB-1 inoculated piglets exhibited no obvious clinical symptoms or macroscopic lesions. PCV3 displayed a broad histotropism, including the heart, liver, spleen, lung, kidney, brain, lymph nodes, and tonsil, and the lungs and lymph nodes contained a higher quantity of viral genomes compared to that of the other organs. From 7 days after PCV3 DB-1 inoculation, the piglets showed obvious IgG antibody responses against PCV3 rCap-VLPs. The cumulative results demonstrated that PCV3 trend to low pathogenicity.

## 1. Introduction

Porcine circovirus (PCV) is currently recognized as four types (i.e., PCV1, PCV2, PCV3, and PCV4) [1–7], and PCV3 was recently recognized from a swine farm experiencing reproductive failure and porcine dermatitis and nephropathy syndrome- (PDNS-) like clinical signs in the United States in 2015 [3]. The metagenomic sequencing analysis showed that PCV3 has only 48% amino acid identity in the Rep protein and 26% amino acid identity in the Cap protein compared with PCV2 [3].

Since the first report of PCV3 in 2015, almost swine-producing countries in Asia, Europe, and America reported the same disease but highly variable clinical presentations ranging from inapparent to severe respiratory and enteric disease, as well as neurological disorders, multisystemic inflammation, and reproductive failure [8–15]. In China, more than 10 provinces have reported the appearance of this pathogen, and mostly focused on the pathogen appear and cycle through the swine herds [16–19]. Limited by viral isolation and prevalence in both diseased and healthy swine herds, the clinical relevance of PCV3 has being not clear and needs further study.

To investigate the pathogenicity of PCV3 in piglets, in this study, we used a PCV3 isolate (PCV3-China/DB-1/2017, MH286898) to inoculate three-week-old cesarean-derived, colostrum-deprived (CDCD) piglets. Clinical signs, pathological changes, viral load, viral mRNA in the tissue, and antibodies against PCV3 rCap-VLPs were investigated. These results showed that piglets infected with PCV3 DB-1 developed no obvious clinical symptoms or macroscopic lesions. Histological pathological observation showed lymphocyte reduction and a few inflammatory cells infiltration in the lymph nodes, as well as thickened alveolar septum in the lungs. PCV3 replication was detected in the lungs and lymph nodes of piglets using RNA in situ hybridization (RNAscope). The obvious IgG antibody responses trending against the PCV3 rCap-VLPs appeared in five out of nine DB-1 inoculated piglets. In conclusion, our results provide a further explanation for the debatable clinical relevance of PCV3 infection.

## 2. Materials and Methods

### 2.1. Virus

The PCV3 DB-1 isolate (PCV3-China/DB-1/2017, MH286898) used in this study was isolated from the lungs of two 10-day-old piglets in a commercial swine production system in Heilongjiang Province, Northeast China, by passaged three times in PK-15 cells refer to previously [20]. The ORF2 sequences of 80 representative PCV3 complete genomes originated from *Sus scrofa* (provided by NCBI) were downloaded for phylogenetic analysis. The consistent mutations in amino acids 24 and 27 of the cap protein are potential molecular markers for the classification of PCV3 [21]. Sequences were aligned using the Clustal X program with preset parameters in Clustal W (Lynnon Co., DNAMAN software). A phylogenic tree was deduced based on ORF2 by an ML method with 1,000 bootstrap replicates by MEGA 5.0.

### 2.2. Animal Challenge

A total of 18 three-week-old CDCD piglets (free of porcine circovirus type 2/3, porcine parvovirus, classical swine fever virus, or pseudorabies virus, confirmed by real-time PCR) were obtained from the Experimental Animal Center at the Veterinary Research Institute (Harbin, China). The piglets were randomly divided into two groups (nine piglets for PCV3 inoculation and another nine piglets for mock infection). Piglets were housed separately in two rooms and kept under biosafety level 2 conditions throughout the experiment. Piglets in the virus-inoculation group were intranasally (i.n.) and intramuscularly (i.m.) challenged with the PCV3 isolate DB-1at 1.18 × 10^5^ genomic copies, respectively. The other nine piglets were used as control and received DMEM with the same manner. The piglets were monitored daily for clinical symptoms and rectal temperatures. Blood samples were periodically collected (0, 7, 10, 14, 17, 21, and 28 DPI) from piglets for PCV3 and serological detection. Three piglets from the PCV3-infected group and negative control group were humanely euthanized at 14, 21, and 28 DPI, respectively. At necropsy, the tissue sections (heart, liver, spleen, lung, kidney, lymph nodes, tonsil, and brain) were fixed in 10% phosphate-buffered formalin for hematoxylin and eosin (H&E), and RNAscope detection or stored at -70°C for virus quantitation.

### 2.3. Real-Time PCR Quantitation of the Viral Load in the Tissues

The total DNA was isolated from each tissue using a Dneasy Blood & Tissue Mini kit (Qiagen) in accordance with the manufacturer's instructions. TaqMan fluorescent quantitative PCR (q-PCR) was performed to determine the PCV3 viral loads in tissues collected at 14, 21, and 28 DPI according to a previous study [22].

### 2.4. Histopathology Examinations and RNA Detection In Situ Hybridization (ISH)

Tissue samples were fixed in 10% phosphate-buffered formalin, embedded in paraffin, cut into 4 *μ*m sections, and stained with H&E according to the standard procedure. ISH-RNA was performed using RNAscope® 2.5 HD Reagent Kit (Advanced Cell Diagnostics Inc.), targeting the specific nucleotide sequence of the PCV3 viral mRNA (RNAscope® probes, catalog no. 463961 or 530431) for formalin-fixed paraffin-embedded samples. The samples were visualized using an Olympus BX43 bright-field microscope (Olympus Corporation, Tokyo, Japan).

### 2.5. Serology

Serum antibodies against PCV3 were detected using a modified indirect enzyme-linked immunosorbent assay (ELISA) based on PCV3 recombinant virus-like particles (VLPs) [23]. The optical density (OD) was read at 450 nm using an ELISA plate reader (PE, USA). The serum with an OD450 greater than or equal to the cut-off value was considered to be PCV3 antibody positive.

## 3. Results and Discussion

Phylogenetic characterization of ORF2 sequences showed that PCV3 DB-1 is the first isolation of alanine (A) and lysine (K) at positions 24 and 27 within the Cap protein in NCBI database of PCV3 so far. PCV3 DB-1 shared a nucleotide identity of ~98.3-99.8% with PCV3 ORF2 sequences deposited in GenBank® (including 80 representative sequences) (Figure 1(a)). The ORF2 sequence of PCV3 DB-1 exhibited the highest (99.8%) nucleotide identities with MG868940/MN605934/MN605937 and the lowest nucleotide identity (98.3%) with MK033235/MK033209/MG770384/MK568469. Difference analysis of Cap protein amino acid sequences among PCV3 DB-1 and other PCV3 isolates showed five specific amino acid sites, 24 (A/V), 27 (K/R), 77 (S/T), 150 (I/L), and 211 (E/K), respectively (Figure 1(b)). PCV3 is a newly discovered virus, but has been detected retrospectively since 1966 in China [21], 1967 in Brazil [24], 1996 in Spain [13], and 2006 in Thailand [25]. PCV3 has been reported in cases of reproductive failure [26, 27], PDNS, and porcine circovirus-associated disease (PCVAD) in clinical cases [28]. Thus, further studies are necessary to evaluate if the PCV3 DB-1 isolate with A24 and K27 within the Cap might have unique phenotypic traits that can be associated with specific clinical presentations.

In the animal experiment study, the clinical course of the PCV3 DB-1 and mock inoculation in three-week-old cesarean-derived, colostrum-deprived piglets was monitored. During the four weeks of the experiment, there was no significant differences in the rectal temperatures (Figure 2(a)), and body weight gains (Figure 2(b)) between the PCV3 DB-1 and mock inoculated piglets. No obvious macroscopic lesions were found in the lungs, spleens, lymph nodes (mesenteric lymph nodes, inguinal lymph nodes, and submandibular lymph nodes), tonsils, hearts, livers, kidneys, and brains during necropsy at 14, 21, and 28 DPI, respectively.

TaqMan fluorescent quantitative PCR (q-PCR) was performed to determine the viral load in the organs from PCV3-inoculated piglets as previously described [22, 29]. The accurate Ct cut-off was 37 for the detection limit of PCV3 that was positive in the diagnostic samples [22]. The PCV3 viral genome was detected in all of the relevant tissues, including the lung, spleen, lymph nodes (mesenteric lymph nodes, inguinal lymph nodes, and submandibular lymph nodes), tonsil, heart, liver, kidney, and brain; the results demonstrated that PCV3 has a wide range of histotropism (Table 1). Among these tissues, the highest level of the PCV3 viral genome was detected in the lung (Ct 32.1, 10^2.67^ copies/g), lung (Ct 23.3, 10^5.41^ copies/g), and inguinal lymph node (Ct 26.0, 10^4.81^ copies/g) at 14 DPI, 21 DPI, and 28 DPI, respectively. This finding demonstrated that PCV3 can replicate its viral genome more efficiently in the lungs and lymph nodes compared to that of the other tissues. However, PCV3 could not be passaged continuously in PK-15 cells [20], whether PCV3 can be passaged continuously in other cell lines is worth to further investigation.

To further characterize the organ lesions induced by PCV3 DB-1 infection, the lungs and lymph nodes were examined on a microscopic level for histopathological damage. H&E staining of PCV3 DB-1-infected piglets showed lymphocyte reduction, companying by inflammatory cell infiltration in the lymph nodes (Figure 3(a)), as well as epithelial cell proliferation, inflammatory cells infiltration, and thickened alveolar septum in the lungs (Figure 3(c)). Correspondingly, PCV3 replication was detected in the lymph nodes (Figure 4(a)) and lungs (Figure 4(c)) by ISH detection. No obvious pathological damage appeared in the mock-infected piglets (Figures 3(b) and 3(d)), as well as the negative signals in the lymph nodes (Figure 4(b)) and lungs (Figure 4(d)) of the mock-inoculated piglets.

To better understand the humoral immune response elicited by PCV3 DB-1 challenge, the anti-PCV3 antibody titer in the serum samples was assessed by an indirect ELISA based on PCV3 recombinant rCap-VLPs [23]. Throughout the experiment, the IgG antibody response varied among the individuals (Figure 5). Four out of nine PCV3 DB-1-inoculated piglets showed an obvious IgG antibody response from 7 (3/4) or 10 (1/4) DPI. One piglet (1/9) from 14 DPI and the other four piglets (4/9) showed either an absence or mild IgG seroconversion within the 28 days of experimental period. The humoral immune response elicited by PCV3 DB-1 is different from that of PCV3 63911 isolate, which inoculation induced more than one-half of cesarean-derived, colostrum-deprived piglets (5/8) and increased IgM antibody response against the PCV3 Cap protein between 7 and 14 DPI; however, no significant IgG seroconversion was detected in any infected piglet throughout the 28-day study period [20]. The difference between our study and the aforementioned study [20] is that there was a trend in the IgG antibody response against the PCV3 Cap protein. In our study, 5 of nine PCV3 DB-1 inoculated piglets showed an obvious trend in the IgG antibody response. The indirect ELISA method used in our study based on PCV3 recombinant rCap-VLPs [23, 30] might conserve the conformational epitopes and had the ability to detect IgG antibodies against the conformational epitope of the PCV3. Antibodies against rCap-VLPs of PCV3 that appeared in piglets with a specific immune status may be inflammatory factors that alert immune cells to respond to the viral infection; however, whether these antibodies can neutralize PCV3 requires further investigation.

Since the porcine circovirus (PCV3) was first reported from a swine farm in United States, PCV3 has been detected in swine farms throughout the world. Among those reports, clinical signs produced by PCV3 infection appear to be highly variable: sows characterized by reproductive failure and PDNS-like clinical signs [3]; clinical cases from 3 to 10 week piglets show multisystemic and cardiac inflammation [31]; 4-week-old piglets infected with PCV3 DNA clone develop PDNS-like disease and 40% mortality [32]; 6-week-old CDCD pigs with unremarkable visual clinical performance under experimental conditions [20]; and wild boar infection with PCV3 naturally showed nonpathogenic but highly prevalent (30%) [33]. Since there is an abundance of data indicating that a PCV3 infection can cause different clinical outcomes (different clinical syndromes) or subclinical (absence of symptoms) symptoms in domestic pigs [10, 12, 16, 17, 28, 34–37], PCV3 pathogenicity has become controversial and requires experimental data to reduce this controversial academic issue. In our study, the outcome of PCV3 inoculation to CDCD piglets indicates PCV3 infection cannot induce obvious clinical symptoms and pathological changes. The appearance of clinical symptoms and the severity of the disease may be affected by the immune status of pigs [38, 39], stress factors that cause systemic inflammation [40, 41], or coinfection with other pig pathogens [42, 43]. The cumulative results in our study demonstrated that PCV3 trend to low pathogenicity. Whether the synergy between PCV3 and bacterial/viral coinfections warrants further investigation [44, 45].

In conclusion, piglets inoculated by PCV3 DB-1 isolate with the molecular characterization of 24A and 27K exhibited no obvious clinical symptoms or macroscopic lesions. However, this isolate showed a broad histotropism, and the lungs and lymph nodes contained a higher quantity of viral genomes among the detected organs, as well as the infection induced obvious IgG antibody against PCV3 rCap-VLPs. These results imply that PCV3 DB-1 isolate trends to low pathogenicity to the piglets.

## Figures and Tables

**Figure 1:** Phylogenetic analysis based on the ORF2 sequences of the PCV3 representative sequences (a). The ML tree was reconstructed using MEGA 5.0 with 1,000 bootstrap trials. The values along the branches represent bootstrap values. Difference analysis of the amino acid sequences of Cap protein of the PCV3 isolates (b). Yellow-shaded amino acids represent a difference in amino acid sequence of the PCV3 isolates.

**Figure 2:** Rectal temperatures (a) and body weight gains (b) of the PCV3-inoculated and mock-inoculated piglets. No significant differences in rectal temperatures and body weight gains of the piglets were found between the PCV3-inoculated and mock-inoculated groups during the four weeks of the experiment. Mean ± SD (error bars) temperatures or body weight gain are shown.

**Figure 3:** Histopathological lesions of the lymph nodes (a, b) and lungs (c, d) from PCV3- and mock-inoculated piglets. The piglets infected with the PCV3 DB-1 isolate showed a small number of lymphocyte reduction and inflammatory cell infiltration in the lymph nodes (a), and epithelial cell proliferation, inflammatory cells infiltration, and thickened alveolar septum in the lungs (c). No obvious pathological lesions were observed in the lymph nodes (b) and lungs (d) of the mock-inoculated piglets.

**Figure 4:** RNAscope in situ hybridization of the lymph nodes (a, b) and lungs (c, d) from PCV3- and mock-inoculated piglets. The PCV3 DB-1 infected piglets showed positive signals in the lymph nodes (a) and lungs (c). No obvious positive signals were observed in the lymph nodes (b) or lungs (d) of the mock-inoculated piglets.

**Figure 5:** Detection of IgG antibodies against PCV3 rCap-VLPs antigens. IgG antibody responses (mean OD450 values) detected by PCV3 rCap-VLPs indirect ELISA in three-week-old CDCD piglets (*n* = 18) following experimental inoculation with PCV3 isolate DB-1 or negative control (0-14 dpi, *n* = 9; 14-21 dpi, *n* = 6; 21-28 dpi, *n* = 3) over the course of the infection. Mean ± SD (error bars) of the specific antibodies are shown.

**Table 1:** The dynamics of virus distribution in the organs of PCV3- and mock-inoculated piglets.

Ct values (copies/g)		14 DPI	21 DPI	28 DPI	Control
Tissue	Heart	32.2 (10^2.65^)	29.7 (10^3.51^)	31.0 (10^3.09^)	—
	Liver	32.4 (10^2.64^)	27.2 (10^4.29^)	28.9 (10^3.79^)	—
	Spleen	32.2 (10^2.65^)	26.6 (10^4.51^)	27.7 (10^4.14^)	—
	Lung	32.1 (10^2.67^)	23.3 (10^5.41^)	26.3 (10^4.53^)	—
	Kidney	33.1 (10^2.40^)	29.7 (10^3.51^)	30.3 (10^3.38^)	—
	Brain	32.4 (10^2.64^)	30.4 (10^3.37^)	30.2 (10^3.39^)	—
	ILN	33.6 (10^2.36^)	25.8 (10^4.86^)	26.0 (10^4.81^)	—
	SLN	33.2 (10^2.40^)	27.5 (10^4.19^)	26.6 (10^4.51^)	—
	MLN	33.6 (10^2.37^)	28.3 (10^3.94^)	27.9 (10^4.10^)	—
	Tonsil	33.1 (10^2.40^)	31.3 (10^3.01^)	30.4 (10^3.37^)	—

MLN: mesenteric lymph nodes, ILN: inguinal lymph nodes, SLN: submandibular lymph nodes; —: higher than Ct cut-off value; each number represents the average Ct values (copies/g) generated from at least three times detection.

## Data Availability

The datasets used and/or analyzed during the current study are available from the corresponding author on reasonable request.
